The article "Effect of Polyethylene Cover for Preventing Corneal Injury in Critically Ill Patients: A Meta-Analysis" was retracted in 2023. Reasons: unreliable results or conclusions; concerns about the data; concerns about the peer review; concerns about the citations.

# Effect of Polyethylene Cover for Preventing Corneal Injury in Critically Ill Patients: A Meta-Analysis

**DOI:** 10.1155/2022/6578229

**Published:** 2022-01-28

**Authors:** Tao Li, Huijuan Zhou

**Affiliations:** ^1^Department of Ophthalmology, The First Affiliated Hospital of Soochow University, Suzhou of Jiangsu Province, Suzhou 215006, China; ^2^Department of Internal Medicine, The First Affiliated Hospital of Soochow University, Suzhou of Jiangsu Province, Suzhou 215006, China

## Abstract

**Objective:**

Polyethylene cover has been proved to be an effective method in protecting corneal, but its advantage compared to other conventional methods is still unclear. Our study is aimed at assessing clinical effects of polyethylene cover versus other methods in the prevention of corneal injury for critically ill patients.

**Methods:**

We searched randomized controlled trials comparing polyethylene cover versus other methods for critically ill patients through the databases of PubMed, Embase, Web of Science, and China National Knowledge database. Forest plots and funnel plots were also performed on the included articles. Results were expressed as risk ratio (RR) with 95% confidence intervals.

**Results:**

Eight studies were eventually identified. The incidence of corneal injury in the polyethylene cover group was lower than that in the eye drops group (RR = 0.24, 95% CI (0.12, 0.45), *P* < 0.0001) but had no significant difference when compared to the eye gel group (RR = 0.42, 95% CI (0.13, 1.34), *P* = 0.14) and the eye ointment group (RR = −0.61, 95% CI (0.23, 1.59), *P* = 0.31).

**Conclusion:**

This study showed that polyethylene cover, eye gel, and eye ointment had an equal effect for preventing corneal injury in critically ill patients, and the effect of eye drops was relatively low. However, there were other intervention methods that had not been compared due to the small number of articles; further studies should be performed to assess which method was the best practice method.

## 1. Introduction

The cornea is an epithelial tissue without vascular distribution, stratum corneum, and secretory glands. It relies on tears to maintain moisture and transport oxygen and nutrients for oxygen metabolism. Eyelid closure and blinking will produce tears and transport them to the cornea to prevent the tears from evaporating [1]. The body resistance of patients is seriously reduced [2, 3]. At the same time, some patients have abnormal eyelid closure, which leads to a high incidence of eye complications [4, 5]. Serious cases can develop into severe corneal injury, resulting in permanent vision defects or blindness, affecting the normal life of patients [6–8].

The article "Effect of Polyethylene Cover for Preventing Corneal Injury in Critically Ill Patients: A Meta-Analysis" was retracted in 2023. Reasons: unreliable results or conclusions; concerns about the data; concerns about the peer review; concerns about the citations.

It had been reported that the incidence of cornea injury in patients admitted to intensive care unit (ICU) for 2-7 days was 20%-40% [9]. Therefore, nurses should take effective nursing measures to prevent the occurrence of corneal injury in ICU patients. Clinically, there are several therapies to prevent cornea injury: polyethylene cover, eye drops, eye gel, eye ointment, and labrilube [10, 11].

Although some studies had confirmed that polyethylene cover can prevent corneal injury in patients with decreased or disappeared blink reflex, most of them were small sample studies with weak persuasion [12, 13]. The intervention methods of the control group in the study were quite different, and the conclusion was also different when polyethylene cover therapy compared with other therapy [14–16].

This study intended to use meta-analysis to combine the results of different research, compared the incidence of corneal injury with different intervention methods, and aimed to explore the effect of polyethylene cover in preventing corneal injury in critically ill patients.

## 2. Methods

### 2.1. Literature Search Strategy

Systematic searches have been carried out in PubMed, Embase, Web of Science, and China National Knowledge database up to October 2021, with the following keywords: (1) polyethylene cover, (2) corneal injury, and (3) critically ill patients; all these words were combined using the Boolean operator “and/or.” A comprehensive search of the literature was carried out, which had no limitation on the publishing language or publishing status. In order to achieve maximal sensitivity of the search result, we also check the reference of the searched articles to look for other relevant studies that were not found in our search strategy.

### 2.2. Study Selection

We included articles that met the following inclusion criteria:

1. Researches comparing patients receiving polyethylene cover and other treatment
2. Outcome indexes included the incidence of corneal injury or keratitis
3. Full-text articles could be implemented

We excluded studies meeting the following exclusion criteria:

1. Researches on other treatments not included polyethylene cover
2. Articles that were only available as abstracts or letters were not considered
3. Study lacking available data

### 2.3. Data Extraction and Quality Assessment

Two investigators independently reviewed the full text of eligible studies and extracted data using a prespecified data collection form, including the following information: first author's name, language, patient's age and gender, country of origin, year of publication, type of study, sample size, the study duration, and primary conclusion. The Cochrane bias risk assessment tool was used to evaluate the overall methodological quality of included studies.

The article "Effect of Polyethylene Cover for Preventing Corneal Injury in Critically Ill Patients: A Meta-Analysis" was retracted in 2023. Reasons: unreliable results or conclusions; concerns about the data; concerns about the peer review; concerns about the citations.

### 2.4. Statistical Analysis

RevMan 5.4 software was used for meta-analysis. The chi-square test and *I*^2^ were used to detect the heterogeneity among studies. The *I*^2^ value exceeded 25%, 50%, and 70%, indicating low, moderate, and high heterogeneity among studies, respectively. It was generally believed that *I*^2^ ≥ 50% indicates substantial heterogeneity. The fixed-effects model was used to analyze for homogeneous studies; otherwise, a random-effects model was performed to calculate the pooled results.

## 3. Results

### 3.1. Search Process

A total of 475 studies were screened through the electronic search procedure. Sixty-two studies met the inclusion criteria after a careful reading of the full articles. We further excluded 54 studies based on the study design, insufficient data, or improper literature type. After screening, 8 papers were included in this meta-analysis [17–24]. A flow diagram illustrating the searching procedure and exhibiting the inclusion and exclusion criteria is displayed in Figure 1.

### 3.2. Characteristics of Included Studies

Two authors (Li and Zhou) systematically collect data from all selected studies by using standardized data extraction tables, including the first author, language, year of publication, authors' country, sample size, patient's characteristics (age and gender), duration of research, and primordial conclusion.  Table 1 summarizes the basic characteristics of included studies, and Table 2 provides a detailed summary of patients' clinical baseline information and primary conclusion of studies. These studies contained 8 RCTs that involved a total of 580 patients, of which 288 received polyethylene cover treatment and 292 received control treatment (drops, gel, or ointment).

### 3.3. Results of Quality Assessment

Bias risk assessment was conducted at the study level, and methodological quality assessment was assessed using the Cochrane bias risk assessment tool. Through the author's subjective judgment after reading the full text, high risk of performance bias and reporting bias was found in two different studies (Figure 2).  Figure 3 summarizes the risk of bias for each included study.

### 3.4. Results of Heterogeneity Test

To analyze the difference of incidence of corneal injury between polyethylene cover therapy and eye drop therapy, we performed a pooled analysis based on heterogeneity analysis. The risk ratio (RR) was 0.24 with 95% CI (0.12, 0.45), while the *P* value of overall effect was <0.001, and no significant heterogeneity among included studies (*P* = 0.41, *I*^2^ = 0%) (Figure 4). The result proved that the incidence of corneal injury in the polyethylene cover group was significantly lower than that in the eye drops group.

The article "Effect of Polyethylene Cover for Preventing Corneal Injury in Critically Ill Patients: A Meta-Analysis" was retracted in 2023. Reasons: unreliable results or conclusions; concerns about the data; concerns about the peer review; concerns about the citations.

Similarly, a meta-analysis for the difference of incidence of corneal injury between polyethylene cover therapy and eye gel therapy was conducted. Incidence difference was analyzed by the fixed-effects model. The risk ratio was 0.42 with 95% CI (0.13, 1.34) (Figure 5, *P* value of overall effect was 0.14, *I*^2^ = 37%). No significant difference of the incidence of corneal injury between the polyethylene cover group and the eye gel group was found.

In the evaluation of difference of incidence of corneal injury between polyethylene cover therapy and eye ointment therapy, 3 articles were included. The risk ratio was -0.61 with 95% CI (0.23, 1.59) (*P* = 0.31, fixed-effects model, Figure 6), and the included articles were homogeneous (*P* = 0.36, *I*^2^ = 1%). It demonstrated that the incidence of corneal injury between the polyethylene cover group and the eye ointment group had no significant difference.

### 3.5. Publication Bias

To assess for any evidence of publication bias among the included studies, funnel plots for all three models were performed. The funnel plot was visually checked, and the shape was relatively asymmetric (Figure 7), but Egger's test was nonsignificant (A, *P* = 0.304; B, *P* = 0.208; C, *P* = 0.367), which indicated that no obvious publication bias existed in our meta-analysis.

## 4. Discussion

Patients in ICU are often critically ill and rely heavily on detection, imaging, and drug treatment [25]. Nursing practice is essential in these units, focusing on providing patients with urgent needs while preventing potential complications [26, 27]. There are many risk factors to weaken the mechanism of eye protection in coma patients in ICU, which are prone to eye diseases [28, 29]. The routine eye care plan is to use eye drops in the daytime and eye ointment to close the eyelids at night, but the effect of clinical intervention is not ideal [30, 31].

Polyethylene cover is a kind of airtight material; its main function is to form a closed cavity around the eyes, prevent the evaporation of tears to keep local moisture, prevent dry eye surface, and effectively protect the eyes of patients [13, 23]. At the same time, it can replace the mechanical barrier of eyelid, prevent foreign body from entering, and prevent physical, chemical, and biological damage [24, 32].

In our study, patients were randomly divided into 4 groups (eye hygiene, eye gel, eye drops, and polyethylene cover). The results showed that the polyethylene cover group was more effective than the control group in reducing the risk of occurrence of corneal injury [16]. In one randomized controlled trial by Kocaçal et al. [30], the control group received only carbomer eye drops while the intervention group received both carbomer eye drops and polyethylene covers; the authors found that carbomer eye drops, when used in combination with polyethylene covers, were effective in managing exposure keratopathy.

The article "Effect of Polyethylene Cover for Preventing Corneal Injury in Critically Ill Patients: A Meta-Analysis" was retracted in 2023. Reasons: unreliable results or conclusions; concerns about the data; concerns about the peer review; concerns about the citations.

Eight studies involving 580 critically ill patients were included in this meta-analysis. Four studies reported the incidence of corneal injury between polyethylene cover therapy and eye drops therapy; meta-analysis showed that the incidence of corneal injury in the polyethylene cover group was significantly lower than those in the eye drops group (*P* < 0.001). Three studies reported the incidence of corneal injury between polyethylene cover therapy and eye gel therapy, and the result showed no significant difference between two groups (*P* = 0.14). Another three articles compared the incidence of corneal injury between polyethylene cover therapy and eye ointment therapy; no statistical difference was found (*P* = 0.31).

Due to the damage of eye protection mechanism, severe patients were more prone to eye complications than ordinary patients. The higher rate of corneal injury should arouse the attention of clinical workers to the eye care needs of severe patients [33, 34]. Our study showed that polyethylene cover had some advantages over eye drops, but no obvious advantage compared with eye gel and eye ointment. Therefore, according to the different conditions of patients, ICU can take into account the effect guarantee of nursing intervention, the comfort of patients, and the workload of nursing staff and selectively use one or more schemes of nursing intervention, so as to achieve the purpose of reducing the eye complications of severe patients [35–37].

In conclusion, this study showed that polyethylene cover, eye gels, and eye ointments were equally effective in preventing corneal injury in critically ill patients, while eye drops were relatively less effective. However, inevitable limitations existed in our meta-analysis; there were still other methods to prevent corneal injury for critically ill patients, such as labrilube and moisture chamber by swimming goggles, but few research compared these two methods with polyethylene cover [25, 38, 39], which method was the optimal practice method that should be further studied.

## Figures and Tables

**Figure 1:** Flow diagram of study selection process.

**Figure 2:** Quality assessment of included studies: low risk (green color), unclear (yellow color), and high risk (red color).

**Figure 3:** Risk of bias summary of included studies.

The article "Effect of Polyethylene Cover for Preventing Corneal Injury in Critically Ill Patients: A Meta-Analysis" was retracted in 2023. Reasons: unreliable results or conclusions; concerns about the data; concerns about the peer review; concerns about the citations.

**Figure 4:** Forest plot: comparison of incidence of corneal injury between polyethylene cover group and eye drops group. RR: risk ratio.

**Figure 5:** Forest plot: comparison of incidence of corneal injury between polyethylene cover group and eye gel group. RR: risk ratio.

**Figure 6:** Forest plot: comparison of incidence of corneal injury between polyethylene cover group and eye ointment group. RR: risk ratio.

**Figure 7:** Funnel plot of publication bias: (a) polyethylene cover versus eye drops; (b) polyethylene cover versus eye gel; (c) polyethylene cover versus eye ointment.

**Table 1:** Description of included studies.

Study	Country	Language	No. patients		Gender (M/F)		Age		Duration of study
			Experimental	Control	Experimental	Control	Experimental	Control	
Cortese 1995	USA	English	30	30	/	/	/	/	/
Koroloff 2004	Australia	English	50	60	33/17	31/29	50.1 ± 18.6	55.1 ± 18.5	7 month
So 2008	China	English	59	57	35/24	37/20	59.4	61.7	20 month
Shan 2010	China	English	29	28	/	/	55.2 ± 18.8	54.5 ± 18.2	/
Baker 2012	Saudi Arabia	English	20	20	/	/	/	/	5 month
Su 2012	China	Chinese	30	30	17/13	15/15	52.8 ± 8.4	53.9 ± 8.9	11 month
Ahmadinejad 2020	Iran	English	41	42	63/19	67/16	44.9 ± 20.6	40.8 ± 18.0	11 month
Khatiban 2021	Iran	English	29	25	19/10	16/9	/	/	8 month

**Table 2:** Clinical baseline information and primary conclusion of studies.

Study	Study design	Patient type	No. patients		Intervention		Conclusion
			Experimental	Control	Experimental	Control	
Cortese 1995	RCT	Critically ill patients	30	30	Polyethylene cover	Methylcellulose lubricating drops every 2 h	Moisture chamber is more effective than lubricating drops in preventing corneal epithelial breakdown in critically ill patients with limited or absent blink reflex
Koroloff 2004	RCT	Semiconscious intensive care patient	50	60	Polyethylene cover	Combining hypromellose drops and Lacri-Lube every 2 h	Polyethylene covers are as effective as HL in reducing the incidence of corneal damage in intensive care patients
So 2008	RCT	Critically ill patients	59	57	Polyethylene cover	1 cm of Duratears ointment every 4 h	Polyethylene cover is found to be equally effective in preventing corneal abrasions when compared with lanolin eye ointment
Shan 2010	RCT	ICU	29	28	Polyethylene cover	Two drops of carboxymethylcellulose drops every 2 h	Polyethylene covers are more effective and more time-saving in reducing the incidence of corneal damage in intensive care patients
Baker 2012	RCT	Ventilated patients in ICU	20	20	Polyethylene cover	One drop of Viscotears (polyacrylic acid viscous gel) every 8 h	The use of polyethylene cover and Viscotears gel were equally effective in prevention of corneal abrasions in critically ill patients
Su 2012	RCT	Critically ill patients	30	30	Polyethylene cover	Artificial eye gels and antibiotic ointment every 4 h	Using polyethylene film for eye care of critically ill patients can effectively prevent eye complications and prevent eye dryness
Ahmadinejad 2020	RCT	Critically ill patients	41	42	Polyethylene cover	2 cm of ointment every 2 h	Polyethylene cover followed by simple eye ointment and eyelid taping were the most effective methods in preventing ocular surface disorders
Khatiban 2021	RCT	Comatose patients	29	25	Polyethylene cover	Artificial teardrops (polyvinyl alcohol or hydroxypropyl methylcellulose)	Polyethylene eye covers significantly reduced the incidence and severity of ocular surface disorders

RCT: randomized controlled trails.

The article "Effect of Polyethylene Cover for Preventing Corneal Injury in Critically Ill Patients: A Meta-Analysis" was retracted in 2023. Reasons: unreliable results or conclusions; concerns about the data; concerns about the peer review; concerns about the citations.

## Data Availability

No data were used to support this study.
